# Application Value of Combined Detection of DCE-MRI and Serum Tumor Markers HE4, Ki67, and HK10 in the Diagnosis of Ovarian Cancer

**DOI:** 10.1155/2022/1533261

**Published:** 2022-06-14

**Authors:** Quanzhi Wang, Hui Dong, Peng Zhou

**Affiliations:** ^1^Department of Pathology, Shouguang People's Hospital, Weifang 262700, Shandong, China; ^2^Department of Imaging, Central Hospital Affiliated to Shandong First Medical University, Jinan 250013, Shandong, China

## Abstract

**Objective:**

To investigate the application value of the combined detection of DCE-MRI and serum tumor markers (HE4, Ki67, and HK10) in the diagnosis of ovarian cancer.

**Methods:**

The clinical data of 40 patients with advanced ovarian cancer (AOC) confirmed by surgery and pathology in our hospital from February 2019 to February 2020 were retrospectively analyzed. All patients received DCE-MRI, the detection of serum tumor markers HE4, Ki67, and HK10, and the combined detection of DCE-MRI and the serum tumor markers (HE4, Ki67, and HK10). The application value of the three detection methods was analyzed.

**Results:**

The number of true positives in the single detection (DCE-MRI detection and the detection of serum HE4, Ki67, and HK10) was notably lower than that in the combined detection. The sensitivity, specificity, and accuracy of the single detection were notably lower compared with the combined detection. The area under the curve in the ROC of the combined detection was notably larger than that of the single detection. The results of the combined detection were better than those of the single detection (*P* < 0.05), with the highest sensitivity of the combined detection.

**Conclusion:**

The combined detection of DCE-MRI and the serum tumor markers (HE4, Ki67, and HK10) can effectively improve the diagnostic accuracy of AOC patients, with high sensitivity and specificity, which has an important diagnostic value in clinic.

## 1. Introduction

Ovarian cancer (OC) is a common gynecological malignant tumor, which refers to the malignant tumor arising in the ovary, with an incidence ranking third (second only to cervical cancer and corpus carcinoma) but the highest mortality rate in gynecological malignant tumors, and a five-year survival rate of less than 29% [1, 2]. In addition, negative emotions, long-term malnutrition, and being overweight are the factors causing the occurrence of OC. It has been reported that the 74% of patients have been in the late stage when diagnosed due to the insidious onset of OC, and the survival rate of patients with advanced ovarian cancer (AOC) has not been significantly improved for nearly 29 years due to the lack of effective treatment for advanced cases at present [3, 4]. Presently, the etiology of OC remains unclear, but most scholars believe that it may be related to gynecological diseases, genetics, fertility factors, environment, hormones, and life factors [5, 6]. Epidemiological studies have shown that people carrying BRCA1 and BRCA2 gene mutations have an OC risk of 53% and 22% who are high-risk groups for OC [7]. Jiang Rong et al. [8] have reported that OC is often asymptomatic in the early stage, and in the late stage, it causes some gastrointestinal symptoms such as abdominal distension, lower abdominal discomfort, and loss of appetite in patients, as well as some manifestations such as anemia and weight loss in some patients. At present, though the pathological examination is the gold standard of OC diagnosis, most patients can hardly accept it because it belongs to invasive examination, which is not conducive to early screening. Therefore, it is of a great significance to find a detection method capable of diagnosing OC early [9].

MRI and detecting serum tumor markers are not only common methods to confirm OC diagnosis clinically but also can further evaluate the recurrence and metastasis of OC [10]. MRI detection can provide an effective reference for the evaluation of curative effects for accurately locating and measuring lesions, but MRI has the shortcomings of slow-imaging speed, long inspection time, and high cost, and the accuracy of MRI alone fails to meet clinical expectations. The detection of serum tumor markers plays an important role in tumor diagnosis, the evaluation of clinical efficacy, and prognosis, but it can easily cause misdiagnosis and missed diagnosis for its unsatisfactory sensitivity and specificity [11]. In addition, the previous literature has reported that MRI has a significant application value in the diagnosis of diseases such as gastric cancer, lung cancer, liver cancer, and tongue cancer [12]. The diagnostic effect of serum tumor markers has also been confirmed in digestive system tumors, peritoneal metastasis of gastric cancer, and pancreatic cancer [13]. However, the combined diagnostic effect of the two has rarely been reported. Therefore, this study used the combined detection of DCE-MRI and the serum tumor markers (HE4, Ki67, and hK10) to provide more evidence for subsequent clinical treatment, summarized as follows.

## 2. Materials and Methods

### 2.1. General Information

The clinical data of 40 AOC patients confirmed by surgery and pathology in our hospital from February 2019 to February 2020 were retrospectively analyzed. This study conformed to the Declaration of Helsinki [14].

### 2.2. Recruitment of Research Subjects

#### 2.2.1. Inclusion Criteria

Inclusion criteria were defined as follows: (1) patients who met the diagnostic criteria of OC in obstetrics and gynecology [15] and were confirmed with OC by pathology and cytology, with the clinical manifestations including vaginal bleeding after menopause, masculine sign, hypogastrium discomfort, emaciation, and weakness; (2) patients who received DCE-MRI scanning within 7 days before surgery; (3) serum tumor markers (HE4, Ki67, and HK10) collected within 7 days before surgery; (4) patients who had the first onset and did not receive the treatments such as radiotherapy and chemotherapy; (5) patients who had no family history of hereditary tumors; and (6) patients who had no history of chronic diseases such as diabetes.

#### 2.2.2. Exclusion Criteria

Exclusion criteria were defined as follows: (1) patients in pregnancy and lactation; (2) patients with metastatic OC; (3) patients complicated with severe heart and lung diseases and severe hepatic and renal insufficiency; (4) patients with other malignant tumors; (5) patients with incomplete clinical, pathological, and imaging data; (6) patients receiving DCE-MRI imaging and detection of serum tumor markers 7 days before surgery; (7) patients complicated with cervical diseases such as cervicitis and hysteromyoma; (8) patients with mental disorders; and (9) patients who were participating in other trials.

### 2.3. Methods

#### 2.3.1. DCE-MRI Detection

Before the examination, the relevant precautions of DCE-MRI detection were explained to patients, including early fasting and water deprivation for more than 6 h and removal of metal items from the body before scanning. With the patients in the supine position, a sandbag was placed on their abdomen to reduce the effect of breathing on imaging results, and scanning was performed with an MRI scanner (manufacturer: Philips Medical Technology Co., Ltd.; model: Achieva 3.0 T). Routine scanning was performed on the patients first with the parameters for cross-sectional FSW (T1WI: TE of 11 ms, TR of 40 ms, scan field of 270  mm ^*∗*^ 270 mm and layer thickness of 5 mm; T2WI: TR of 2550 ms, and layer thickness of 4 mm) and sagittal FSE (T1WI: TR of 3200 ms, TE of 85 ms, scan field of 240  mm ^*∗*^ 240 mm, and layer thickness of 4 mm). Then, the routine scanning was converted to the DCE mode, and the patients were intravenously injected with a paramagnetic contrast agent gadodiamide injection (manufacturer: GE Healthcare Ireland; NMPA approval No.: J20100061; specification: 10 ml: 2.87 g) from the elbow at a dose of 0.1 mmol/kg and an injection rate of 3 ml/s using a high-pressure syringe, followed by the saline flush (20 ml) after injection. The DWI parameters were TR of 4900 ms, TE of 77 ms, scanning field of 370  mm ^*∗*^ 370 mm, and layer thickness of 4 mm. With the b-values taken at 400, 700, and 1100 s/mm^2^, 36 times of images were acquired in total and the acquired MRI images were uploaded to the workstation for processing, while the ADC images were generated automatically. The locations with necrosis, hemorrhage, and cystic lesions were avoided as much as possible.

#### 2.3.2. Detection of Serum Tumor Markers (HE4, Ki67, and HK10)

Fasting venous blood (5 ml) was collected from all patients and put into the centrifuge tubes, and the tubes were placed in a 37 °C environment to promote the coagulation. After the blood was coagulated, it was balanced and then centrifuged and the supernatant obtained was the serum, which was extracted carefully and then packed for standby application. The HE4 and Ki67 levels of the patients were measured by using an automatic biochemical analyzer (manufacturer: Getein Biotech Inc.; model: CM-800), and the serum HK10 was measured by an enzyme-linked immunosorbent assay. All procedures were strictly carried out according to the kit (manufacturer: Shanghai Tongwei Industrial Co., Ltd.) instructions.

#### 2.3.3. Positive Determination Criteria

The patients were positive when HE4 ≥ 140 pmol/L, Ki67 ≥ 50 pg/mL, or HK10 > 1040 ng/L.

### 2.4. Observation Indexes

The number of true positives, false positives, true negatives, and false negatives of DCE-MRI, the detection of serum tumor markers (HE4, Ki67, and HK10), and the combined detection of DCE-MRI and serum tumor markers (HE4, Ki67, and HK10) were compared.

The sensitivity, specificity, and accuracy of DCE-MRI, the detection of serum tumor markers (HE4, Ki67, and HK10), and the combined detection of DCE-MRI and serum tumor markers (HE4, Ki67, and HK10) were compared. Sensitivity = number of true positives/(number of true positives + number of false negatives) ^*∗*^ 100%; specificity = number of true negatives/(number of true negatives + number of false positives) ^*∗*^ 100%; and accuracy = number of accurate diagnosis/total number of patients × 100%.

The diagnostic value of the three modalities was compared by plotting the ROC curve.

### 2.5. Statistical Treatment

All experimental data were statistically analyzed and processed by SPSS21.0 software and graphed by GraphPad Prism 7 (GraphPad Software, San Diego, USA). Enumeration data were tested by the *X*^2^ test and expressed as [*n* (%)], while measurement data were tested by the *t*-test and expressed as ($\bar{x}$ ± *s*). When *P* < 0.05, the differences were statistically significant.

## 3. Results

### 3.1. Statistics of Baseline Data of All Subjects

The statistics of baseline data of all subjects are shown in Table 1.

### 3.2. Comparison of True Positive, False Positive, True Negative, and False Negative between Single Detection and Combined Detection

The number of true positives in the single detection (DCE-MRI detection and the detection of serum HE4, Ki67, and HK10) was notably lower than that in the combined detection. See Table 2.

### 3.3. Comparison of Sensitivity, Specificity, and Accuracy between Single Detection and Combined Detection

The sensitivity, specificity, and accuracy of the single detection were notably lower compared with the combined detection, as demonstrated in Table 3.

### 3.4. Area under the Curve of Single Detection and Combined Detection in the ROC

The area under the curve in the ROC of the combined detection was notably larger than that of the single detection, as shown in Figure 1.

### 3.5. Comparison of the Area of Each Index, Standard Error^a^, Progressive Sig.^b^, And Progressive 95% Confidence Interval

The results of the combined detection were better than those of the single detection (*P* < 0.05), as shown in Table 4.

### 3.6. Comparison of Sensitivity and 1-Specificity

The combined detection had the highest sensitivity, as shown in Table 5.

## 4. Discussion

Epidemiological studies have shown that OC is a common gynecological malignancy second only to breast cancer. Although the incidence of OC is lower than that of breast cancer, it has caused the most gynecological cancer-related deaths, with an annual OC incidence of 190,000 new cases and a mortality rate of 113,000 worldwide [16]. Mitamura Takashi et al. [17] have stated that OC, the 7th most common cancer worldwide, is the 5th most common cause of cancer deaths in women, second only to lung, breast, colorectal, and pancreatic cancer, accounting for more than 2% of all cancers in women. According to statistics, the OC incidence has increased at an annual rate of 0.1% for nearly 20 years, and women have a 1.49% chance of developing OC in their lifetime [18]. OC has no specific symptoms in the early stage, and the optimal treatment period is missed when the disease progresses to the middle or advanced stages, leading to a poor prognosis in some patients. Meanwhile, a previous study has shown that OC has a low 5-year survival rate and is one of the malignant tumors that pose serious threats to the life of women [11]. Therefore, this study aimed to investigate a rapid, efficient, and simple diagnostic modality to be applied in the diagnosis of OC. In this study, the number of true positives in the single detection (DCE-MRI detection and the detection of serum HE4, Ki67, and HK10) was notably lower than that in the combined detection, suggesting that the combined detection has high efficiency in the diagnosis of OC. The reason is that the injection of the contrast agent before DCE-MRI scanning can effectively enhance the clarity of the lesions and surrounding tissues in the images and also provide vascular permeability at the lesions. Clinically, diseases are judged by the blood supply around the lesions and the blood supply around the malignant tumors is abundant with strong blood flow, so the accuracy of DCE-MRI for OC is enhanced. HE4 belongs to the family of orotate tetrasulfide core proteins and is highly expressed in tumors such as OC and endometrial cancer. Ki67 is a nuclear protein encoded by the MKI-67 gene, and its levels in case reports are closely related to the differentiation, invasion, metastasis, and prognosis of many tumors [19]. HK10, a serine protease, has been confirmed in biological experiments to be highly expressed in OC tissues and closely related to the prognosis of OC [15]. Serum tumor marker (HE4, Ki67, and HK10) assays alone cannot accurately determine EC because several factors can affect the serum indices (for example, patients have bacterial infection and other inflammation), so they should be used in combination with DCE-MRI. The combined detection of DCE-MRI and serum tumor markers (HE4, Ki67, and HK10) can give full play to the advantages of diagnosis, with better results when compared with the single detection.

In addition, DCE-MRI can also detect the molecular state of the lesions and surrounding cells, in which malignant tumor cells mostly have fast molecular motion and high density, with high signal intensity in the DCE-MRI imaging process. Thus, DCE-MRI can identify OC clinically. As a new tumor marker, serum HE4 has been reported to be more valuable for the diagnosis of OC in many studies [16]. Trabert Britton et al. [16] included 15 articles to analyze the role of HE4 in the diagnosis of OC by meat and found that HE4 had a high diagnostic value for OC (AUC = 0.89, *Q* = 85.21). Schüler-Toprak Susanne et al. [18] have pointed out that Ki67 is widely used in pathological immunohistochemistry to indicate the activity of cell proliferation, playing a role in maintaining the stability of DNA structure during mitosis. Hao Liang et al. [20] have found that HK10 genes and proteins are highly expressed in OC tissues, suggesting that HK10 may be used for the diagnosis and prognosis of OC and even related to the 5-year survival rate of OC after surgery. In this study, the sensitivity, specificity, and accuracy of the single detection were notably lower than those of the combined detection, suggesting that the single detection can easily cause missed diagnosis and misdiagnosis, while the combined detection has a higher diagnostic accuracy and can effectively avoid the occurrence of missed diagnosis and misdiagnosis. At the same time, the area under the curve in the ROC of the combined detection was notably larger than that of the single detection, with the highest sensitivity of the combined detection (*P* < 0.05), confirming that the combined detection has more advantages and a higher diagnostic value than the single detection. The study has some inadequacies. Firstly, due to the limitations of relevant conditions, this study has a small sample size and limited sample source and lacks representation. Secondly, there is inherent selection bias in retrospective studies, such as the different skills of staff in DCE-MRI examination and preoperative pathological examination. Finally, this study has not included patients from other provinces, so the results may be affected by regional culture, which also affects the final results of the clinical trial to a certain extent. Therefore, it is necessary to further improve the research program, increase the sample size, and carry out multicenter studies to obtain more accurate conclusions.

In conclusion, performing the combined detection of DCE-MRI and serum tumor markers (HE4, Ki67, and HK10) to OC patients can effectively improve the diagnostic accuracy rate and has higher sensitivity and specificity, which provides a new diagnostic assay in clinic and promotes the continuous progression of clinical diagnostic in a comprehensive and systematic manner.

## Figures and Tables

**Figure 1:** Area under the curve of the single detection and the combined detection in the ROC.

**Table 1:** Statistics of baseline data of all subjects.

Items	*N*	Proportion (%)
Average age ($\bar{x}$ ± *s*, yrs)	48.00 ± 5.04	—
BMI ($\bar{x}$ ± *s*, kg/m^2^)	20.08 ± 0.69	—

Menopause		
Yes	32	80.00%
No	8	20.00%

FIGO staging (n)		
I	6	15.00%
II	14	35.00%
III	16	40.00%
IV	4	10.00%

Symptoms		
Abdominal pain/distension	27	67.50%
Vaginal bleeding	5	12.50%
Frequent urination/constipation	5	12.50%
Menstruation changes	3	7.50%

Histologic types		
Ovarian serous carcinoma	27	67.50%
Mucinous carcinoma	4	10.00%
Clear-cell carcinoma	3	7.50%
Endometrioid carcinoma	3	7.50%
Others	3	7.50%

Occupation		
Teachers	9	22.50%
Civil servants	7	17.50%
Accountants	11	27.50%
Individual operators	10	25.00%
Others	3	7.50%

Family income		
≥3000 yuan/(month/person)	25	62.50%
<3000 yuan/(month/person)	15	37.50%

Education		
University	20	50.00%
Middle school	11	27.50%
Primary school	9	22.50%

Nation		
Han	32	80.00%
Others	8	20.00%

Residence		
Urban area	27	67.50%
Rural area	13	32.50%

**Table 2:** Comparison of true positive, false positive, true negative, and false negative between single detection and combined detection (*n* (%)).

Detection methods	True positive (*n*)	False positive (*n*)	True negative (*n*)	False negative (*n*)
DCE-MRI	28 (70.00%) ^*∗*^	4 (10.00%)	5 (12.50%)	3 (7.50%)
Detection of serum HE4, Ki67, and HK10	24 (60.00%)^#^	5 (12.50%)	4 (10.00%)	7 (17.50%)^##^
Combined detection	36 (90.00%)	1 (2.50%)	2 (5.00%)	1 (2.50%)

*Note.* ^*∗*^ An obvious difference in the number of true positives between DCE-MRI and the combined detection (*x*^2^ = 5.000, *P* < 0.05). # indicates an obvious difference in the number of true positives between the combined detection and the detection of serum HE4, Ki67, and HK10 (*x*^2^ = 9.600, *P* < 0.05). ## indicates an obvious difference in the number of false negatives between the combined detection and the detection of serum HE4, Ki67, and HK10 (*x*^2^ = 5.000, *P* < 0.05).

**Table 3:** Comparison of sensitivity, specificity, and accuracy between the single detection and the combined detection.

Detection methods	Sensitivity (%)	Specificity (%)	Accuracy (%)
DCE-MRI	90.32	55.56	28 (70.00%)
Detection of serum HE4, Ki67, and HK10	77.42	44.44	24 (60.00%)
Combined detection	97.29	66.67	36 (90.00%)

**Table 4:** Comparison of the area of each index, standard error^a^, progressive Sig.^b^, and progressive 95% confidence interval.

				Progressive 95% confidence interval	
Detection variables	Area	Standard error^a^	Progressive Sig.^b^	Lower limit	Upper limit
DCE-MRI	0.726	0.083	0.015	0.564	0.887
Detection of serum HE4,Ki67, and HK10	0.602	0.091	0.273	0.424	0.779
Combined detection	0.876	0.061	<0.001	0.757	0.995

**Table 5:** Comparison of sensitivity and 1-specificity.

Detection variables	Positive^a^ if greater than or equal to	Sensitivity	1-specificity
DCE-MRI	−1.0000	1.000	1.000
	0.5000	0.714	0.263
	2.0000	<0.001	<0.001

Detection of serum HE4, Ki67, and HK10	−1.0000	1.000	1.000
	0.5000	0.571	0.368
	2.0000	<0.001	<0.001

Combined detection	−1.0000	1.000	1.000
	0.5000	0.857	0.105
	2.0000	<0.001	<0.001

## Data Availability

Data used to support the findings of this study are available on reasonable request from the corresponding author.
